The article "Classification of Artistic Styles of Chinese Art Paintings Based on the CNN Model" was published in 2022. Journal: Comput Intell Neurosci.

# Classification of Artistic Styles of Chinese Art Paintings Based on the CNN Model

**DOI:** 10.1155/2022/4520913

**Published:** 2022-08-30

**Authors:** Bingquan Chen

**Affiliations:** Department of Tradition Chinese Painting, Xi'an Academy of Fine Arts, Xian, Shaanxi 710000, China

## Abstract

People's appreciation needs of Chinese paintings have gradually increased. The research on automatic classification and recognition of Chinese painting artistic style and its authors have great practical value. This study presents a Chinese painting classification algorithm with higher classification accuracy and better robustness. Using a convolutional neural network (CNN) to extract the features of Chinese painting, the image features of Chinese painting are extracted by fine-tuning the pretrained VGG-F model. The mutual information theory is introduced into embedded machine learning, so that the embedded principle is affected by feature selection and feature importance. An embedded classification algorithm based on mutual information is proposed, and Chinese painting is classified.

## 1. Introduction

In the field of Chinese painting feature extraction and classification, there have been a lot of related research studies [1–7]. With the improvement of living standards, people's pursuit of spiritual life is getting higher and higher, and the appreciation demand for Chinese painting is also gradually increasing. A large number of digital Chinese paintings have appeared on the Internet or in digital museums, but how to effectively use and manage these paintings has become an urgent problem to be solved [5–8]. Therefore, the research on automatic classification and recognition of Chinese painting artistic style and its authors has great practical value. The existing literature adopts the traditional feature extraction method to extract the features of Chinese painting, and the obtained features are relatively single and one-sided. In addition, the existing literature does not deal with the extracted features and directly uses the features for classification, without considering the relationship between features and categories and the influence of feature importance on the classification results.

The DEFC (data embedding framework for classification) [9–15] takes the relevant features obtained through the selective conversion of data samples as the input of the algorithm. Although it is much improved than the existing algorithm, it does not consider the influence of feature importance on the calculation of similar features between objects in the process of calculating similar features between objects, resulting in the restriction of classification results.

The article "Classification of Artistic Styles of Chinese Art Paintings Based on the CNN Model" was published in 2022. Journal: Comput Intell Neurosci.

In view of this, this paper uses a convolutional neural network (CNN) to extract the features of Chinese painting, and the obtained features are more comprehensive and detailed. In order to solve the problems mentioned above, this study extracts the image features of Chinese paintings by fine-tuning the pretrained VGG-F model, introduces the mutual information theory into embedded machine learning, makes the embedded principle affected by feature selection and feature importance, proposes an embedded classification algorithm based on mutual information, and classifies Chinese paintings.

## 2. Classification Model of Chinese Paintings

### 2.1. Fundamental Theory

The DEFC embedded mapping framework [9–15] follows the principle of “friendship is close, hostility is far,” and it introduces two parameters, *C*_*F*_ and *E*_*D*_, to control the embedding process; then,

(1) $$\begin{array}{c} C_{F}=\sum_{i,j=1}^{n}d_{F}\left(X_{i},X_{j}|W_{ij}\right), \end{array}$$

(2) $$\begin{array}{c} D_{E}=\sum_{i,j=1}^{n}d_{E}\left(X_{i},X_{j}|W_{ij}\right), \end{array}$$

where **X**_*i*_ and **X**_*j*_ are the *i*th and *j*th objects in the dataset **X**; *C*_*F*_ and *D*_*E*_ represent the intraclass object distance and the interclass object distance in the dataset **X** under the influence of weight parameters, respectively; *d*_*F*_ is the function of calculating the distance between objects of the same type; *d*_*E*_ is the function of calculating the distance between objects of different types; **W**_*ij*_ is the weight parameter obtained by calculating the similarity between objects **X**_*i*_ and **X**_*j*_; *n* is the total number of objects in the dataset.

The DEFC algorithm mainly includes 3 modules. The first module is a data preprocessing module, including 5 optional processes, namely, scaling, centering, normalization, principal component analysis, and whitening. The second module is the relevant feature calculation module; it calculates the correlation features between objects through the original dataset or the preprocessed dataset and performs the above data preprocessing on the calculated correlation features again to obtain the correlation feature matrix RX. The correlation feature captures the mutual influence between samples, which is beneficial to further discovering the nonlinear structure between the data. Since the dimension of the correlation feature matrix is related to the number of samples and has nothing to do with the feature dimension, dimensionality reduction is achieved when the number of samples is much smaller than the feature dimension. The third module is the embedded computing module, which solves *C*_*F*_ is the smallest or *D*_*E*_ is the largest to get the mapping matrix **P**, and then, **X**_final_=**X**_*R*_**P** is calculated by the matrix transformation **X**_final_, that is, the new dataset after the mapping transformation of the original dataset.

The article "Classification of Artistic Styles of Chinese Art Paintings Based on the CNN Model" was published in 2022. Journal: Comput Intell Neurosci.

Another fundamental theory in this study is mutual information theory (MIT) [16–26]. In 1948, Shannon proposed that “information is something used to remove random uncertainty.” Information entropy refers to the probability of a certain information appearing, and the greater the uncertainty of the variable, the greater the information entropy. Information can be measured by information entropy. Among them, the self-information and its mean can measure the information and the amount of information contained in the information set itself. The mutual information and its mean can measure the information and the amount of the information supplied by each other between sets of information.

Mutual information describes the correlation between two variables and can be used to measure the correlation between features and classification results. To calculate the mutual information of variables *X* and *Y*, first, obtain their respective probability distributions *p*(*x*), *p*(*y*) and the joint probability distribution *p*(*x*, *y*). According to *H*=−∑_*i*=1_^*m*^*P*_*i*_*lbP*_*i*_, the information entropy *H*(*X*) and *H*(*Y*) of variables *X* and *Y* and the joint information entropy *H*(*X*, *Y*) of variables *X* and *Y* can be calculated, where *H* represents the information entropy of the feature, *P*_*i*_ is the probability when the feature takes the *i*th eigenvalue, and *m* is the number of all different eigenvalues.

The mutual information between *X* and *Y* is

(3) $$\begin{array}{c} I\left(X;Y\right)=H\left(X\right)+H\left(Y\right)-H\left(X,Y\right). \end{array}$$

### 2.2. Feature Extraction

In recent years, deep learning imitates the mechanism of the human brain, combines low-level features, obtains high-level features that represent the distributed features of data, and is widely used in object recognition, tracking, and other aspects. The traditional CNN is generally used directly for image classification. This study proposes to take advantage of the enormous advantages of the CNN in feature extraction. Compared with explicit feature extraction, more detailed feature data can be obtained for Chinese paintings in extracting digital features.

Based on the CNN theoretical framework, this study fine-tunes the VGG-F model pretrained on the ImageNet dataset to extract the image features of Chinese paintings. The model is a feed-forward neural network with 5 convolutional layers and 3 fully connected layers. The model adjusts the input image to 224*∗*224 pixels and obtains a 4096-dimensional feature vector.

The article "Classification of Artistic Styles of Chinese Art Paintings Based on the CNN Model" was published in 2022. Journal: Comput Intell Neurosci.

Using the VGG-F model pretrained on natural images is feasible to extract features from Chinese paintings. First, art comes from life, and the painter completes the work through the analysis and understanding of all things in nature. Chinese painting is an artistic reprocessing of natural scenes and another embodiment of a natural image. Second, the deep structure of the VGG-F model can extract complex structures from rich perceptual information and build intrinsic representations in the data. More than 10 million natural images are participating in training; the extracted features will directly or indirectly contain feature information similar to Chinese paintings; this way, helpful information for feature extraction of Chinese paintings can be learned. Finally, although, the number of Chinese paintings in the training dataset in this study is not enough to complete the training of the VGG-F model. But this study adds it as a primer to the VGG-F model; the model is fine-tuned so that the features extracted by the model can better express the artistic style of Chinese painting.

### 2.3. Mutual Information-Based Data Embedded Classification Algorithm

Solve the problem that the DEFC algorithm cannot reflect the influence of feature importance on the relationship between computational objects, resulting in restricted classification results. This study introduces mutual information theory into embedded machine learning. A mutual information-based data embedded classification algorithm is proposed. This algorithm calculates the mutual information between each feature vector and the classification category vector. Determine the feature importance and select features with mutual information value greater than zero to form a new dataset to participate in the classification calculation. Therefore, the classification of Chinese paintings is affected by feature selection and feature importance under the embedded principle of “friendship is close, hostility is far.”

Therefore, formulas (1) and (2) become

(4) $$\begin{array}{c} C_{F}=\sum_{i,j=1}^{n}d_{F}\left(X_{i},X_{j}|W_{ij},T_{\text{Featrure}}\right),\\ D_{E}=\sum_{i,j=1}^{n}d_{E}\left(X_{i},X_{j}|W_{ij},T_{\text{Featrure}}\right), \end{array}$$

where *C*_*F*_ and *D*_*E*_ represent the intraclass object distance and the interclass object distance of dataset **X** under the influence of weight and feature importance, respectively; *d*_*F*_ is the function of calculating the distance between objects of the same type; *d*_*E*_ is the function of calculating the distance between objects of different types; **W**_*ij*_ is the weight parameter obtained by calculating the similarity between objects **X**_*i*_ and **X**_*j*_; **T** feature represents the feature and its feature importance.

The article "Classification of Artistic Styles of Chinese Art Paintings Based on the CNN Model" was published in 2022. Journal: Comput Intell Neurosci.

The image features of paintings are extracted by fine-tuning the pretrained VGG-F model, and similar feature sets between paintings are embedded under the influence of mutual information.

The details of the proposed mutual information-based data embedded classification algorithm are as follows.

Input: training dataset *G* and test dataset G′.

Output: the new training dataset *Z* after the embedded mapping is computed and the test dataset Z′.

Its specific process is as follows.

**Step 1 .**

Calculate the mutual information value set **I** between each feature vector in the dataset **G** and the classification classes vector **Y**. **I**_*i*_ represents the mutual information value between the feature vector **G**_*i*_ and the classification classes vector **Y**, and its calculation formula is

(5) $$\begin{array}{c} I\left(G_{i};Y\right)=H\left(G_{i}\right)+H\left(Y\right)-H\left(G_{i},Y\right). \end{array}$$

**Step 2 .**

Normalize the mutual information value set **I** to obtain the feature weight set *δ*_*i*_=**I**_*i*_/∑_*i*=1_^*d*^**I**_*i*_, where *d* is the feature dimension of the training dataset **G**.

**Step 3 .**

The calculation formulas of the training dataset **X**, the test dataset **X′,** and the feature weight set ***θ*** after feature selection are **X**={**G**_*i*_*| ***I**_*i*_ > 0}, **X**′={**G**_*i*_′*| ***I**_*i*_ > 0}, *θ*={*δ*_*i*_*| ***I**_*i*_ > 0}, respectively, where **G**_*i*_ and **G**_*i*_′ are the eigenvalue vectors of the *i*th feature of the training dataset **G** and the test dataset **G′**, respectively.

**Step 4 .**

Define the category indicator matrix *L*. Then,

(6) $$\begin{array}{c} L_{ij}=\left\{\begin{array}{cc} 1, & X_{i},X_{j},\;\text{the same objects},\\ -1, & X_{i},X_{j},\;\text{no the same objects},\; \end{array}\right. \end{array}$$

where **X**_*i*_ and **X**_*j*_ are the two objects of the training dataset **X** calculated in Step 3, when the objects **X**_*i*_ and **X**_*j*_ are the same objects, **L**_*ij*_=1; otherwise, **L**_*ij*_=−1.

**Step 5 .**

Calculate the similarity matrix **W** between the objects in the set **X**. Common methods for calculating distance is the dot product method, polynomial kernel function method, Cosine similarity method, Euclidean distance, and Gaussian kernel function. In this study, various similarity algorithms are used to conduct a large number of experimental calculations. Through experiments, it is found that the classification effect is the best when the cosine similarity method is used. In this study, the cosine similarity method is used to calculate the similarity between objects, and the calculation formula of the similarity matrix **W** is

(7) $$\begin{array}{c} W_{ij}=\left|\frac{X_{i}^{\text{T}}X_{j}}{X_{i}X_{j}}\right|, \end{array}$$

where **W**_*ij*_ represents the similarity between the two objects **X**_*i*_ and **X**_*j*_ of the training dataset **X** calculated in Step 3; **X**_*i*_ and **X**_*j*_ are the modulus of the eigenvectors of objects ‖**X**_*i*_‖ and ‖**X**_*j*_‖, respectively.

The article "Classification of Artistic Styles of Chinese Art Paintings Based on the CNN Model" was published in 2022. Journal: Comput Intell Neurosci.

**Step 6 .**

Calculate the similar feature set **S** between the objects in the set **X**, the similar feature set **S′** between the objects in the set **X′** and the objects in the set *X*.

Let **S**_*ij*_=*φ*(**X**_*i*_, **X**_*j*_), where **X**_*i*_ and **X**_*j*_ are the *i*th and *j*th objects of the training dataset ***X***, *φ*(**X**_*i*_, **X**_*j*_) is the similar eigenvalue calculation function of the objects **X**_*i*_ and **X**_*j*_, the matrix **S** is an *n* × *n* dimensional matrix, and *n* is the set **X** number of objects.

Let **S**_*ij*_′=*φ*(**X**_*i*_′, **X**_*j*_), **X**_*i*_′ is the *i*th object in the test dataset **X′**, **X**_*j*_ is the *j*th object in the training dataset ***X***, *φ*(**X**_*i*_′, **X**_*j*_) is the calculation function of similar eigenvalues of objects **X′** and **X**_*j*_, the matrix **S′** is an *n*′×*n* dimensional matrix, *n* and *n*′ are the number of objects in the sets **X** and **X′**, respectively.

This study uses the distance between two objects as their similar feature. When formulas (1) and (2) calculate the distance, the weight of each feature is the same. However, for Chinese painting, each feature expresses different styles differently. Therefore, this study uses the feature weight set *θ* calculated in Step 3 to calculate the weighted feature distance and use it as the similar feature value between each object.

This study calculates the weighted feature distance based on the weighted norm theory.

Let **X**=(**x**_1_,…,**x**_*l*_)^T^, **Y**=(**y**_1_,…,**y**_*l*_)^T^, **w**_1_,…, **w**_*l*_ be a positive real number and satisfy ∑_*h*=1_^*l*^**w**_*h*_=1, then $d\left(X,Y\right)=\sqrt{\sum_{h=1}^{l}w_{h}^{\alpha }{\left(x_{h}-y_{h}\right)}^{2}}$ is the weighted feature distance between **X** and **Y**, where *α* is the feature weight coefficient.

To sum up, the similar eigenvalues of objects **X**_*i*_ and **X**_*j*_ in the training dataset **X** calculated in Step 3 is $S_{ij}=\sqrt{\sum_{k=1}^{m}\theta_{k}^{\alpha }{\left(X_{ik}-X_{jk}\right)}^{2}}$, where **S**_*ij*_ is the similar eigenvalues between objects **X**_*i*_ and **X**_*j*_; *m* is the feature dimension; *θ*_*k*_ is the feature weight of the kth feature; **X**_*ik*_ and **X**_*jk*_ are the eigenvalues of the *k*th feature of the objects **X**_*i*_ and **X**_*j*_, respectively.

The article "Classification of Artistic Styles of Chinese Art Paintings Based on the CNN Model" was published in 2022. Journal: Comput Intell Neurosci.

**Step 7 .**

Calculate the optimal projection matrix **P**.

Take the similar feature set S calculated in Step 6 as the training sample; the set **Z** represents the new dataset generated by the mapping projection of **S**; let **Z** = **SP** represents the mapping transformation from the set **S** to **Z**, where **P** is the projection matrix, **PP**^T^=**I**, and **I** is the unity matrix.

Using the category indicator matrix **L** and similarity matrix **W** calculated in Steps 4 and 5, set the intraclass object distance *C*_F_ and interclass object distance *D*_E_ of set *Z* as

(8) $$\begin{array}{c} C_{F}=\sum_{i,j=1}^{m}\frac{L_{ij}\left(L_{ij}+1\right)}{2}W_{ij}{\left\|Z_{i}-Z_{j}\right\|}^{2},\\ D_{E}=\sum_{i,j=1}^{m}\frac{L_{ij}\left(L_{ij}-1\right)}{2}W_{ij}{\left\|Z_{i}-Z_{j}\right\|}^{2}, \end{array}$$

where **m** is the feature dimension of the set **Z**.

Set up:

(9) $$\begin{array}{c} B^{\prime }=\left[b_{ij}^{\prime }\right],\\ A^{\prime }=\left[a_{ij}^{\prime }\right], \end{array}$$

where

(10) $$\begin{array}{c} b_{ij}^{\prime }=L_{ij}\left(L_{ij}+1\right)W_{ij},\\ a_{ij}^{\prime }=L_{ij}\left(L_{ij}-1\right)W_{ij}. \end{array}$$

Reconstructing formulas (11) and (12) in matrix form, then

(11) $$\begin{array}{c} B^{\prime }=L\cdot \left(L+I_{m\times m}\right)\cdot W, \end{array}$$

(12) $$\begin{array}{c} A^{\prime }=L\cdot \left(L+I_{m\times m}\right)\cdot W, \end{array}$$

where **I**_*m*×*m*_ is an all-one matrix with *m* rows and *m* columns.

Substitute formula (6) into formula (3). Minimizing *C*_F_, then

(13) $$\begin{array}{c} \underset{pp^{\text{T}}=1}{\text{min}}C_{F}=\underset{pp^{\text{T}}=1}{\text{min}}\sum_{i.j=1}^{d}\frac{B_{ij}^{\prime }}{2}Z_{i}-Z_{j}{}^{2}\\ =\underset{pp^{\text{T}}=1}{\text{min}}tr\left(\sum_{i,j=1}^{d}Z_{i}B_{ij}^{\prime }Z_{i}^{T}-\sum_{i,j=1}^{d}Z_{i}B_{ij}^{\prime }Z_{i}^{T}\right)\\ =\underset{pp^{\text{T}}=1}{\text{min}}tr\left(Z\text{diag}\left(B^{\prime }\right)Z^{T}-ZB^{\prime }Z^{\text{T}}\right)\\ =\underset{pp^{\text{T}}=1}{\text{min}}tr\left(Z\left(\text{diag}\left(B^{\prime }\right)-B^{\prime }\right)Z^{\text{T}}\right). \end{array}$$

Substitute formula (7) into formula (4); maximizing *D*_E_, then

(14) $$\begin{array}{c} \underset{pp^{\text{T}}=1}{\text{max}}D_{\text{E}}=\underset{pp^{\text{T}}=1}{\text{max}}\sum_{i,j=1}^{d}\frac{A_{ij}^{\prime }}{2}Z_{i}-Z_{j}^{2}=\\ \underset{pp^{\text{T}}=1}{\text{max}}tr\left(\sum_{i,j=1}^{d}Z_{i}A_{ij}^{\prime }Z_{i}^{\text{T}}-\overset{d}{\underset{i,j=1}{\sum }}Z_{i}A_{ij}^{\prime }Z_{j}^{\text{T}}\right)=\\ \underset{pp^{\text{T}}=1}{\text{max}}tr\left(Z\text{diag}\left(A^{\prime }\right)Z^{\text{T}}-ZA^{\prime }Z^{\text{T}}\right)=\\ \underset{pp^{\text{T}}=1}{\text{max}}tr\left(Z\left(\text{diag}\left(A^{\prime }\right)-A^{\prime }\right)Z^{\text{T}}\right), \end{array}$$

where diag(**B**′) represents the diagonal matrix of matrix **B**′, and diag(**A**′) represents the diagonal matrix of matrix **A**′; then, the Laplacian matrices of matrices **A**′ and **B**′ are, respectively, as

(15) $$\begin{array}{c} B=\text{diag}\left(B^{\prime }\right)-B^{\prime },\\ A=\text{diag}\left(A^{\prime }\right)-A^{\prime }. \end{array}$$

Because the matrix **L** and the **W** are the symmetric matrices, the matrices **A**, **B**, **ZAZ**^*T*^, and **ZBZ**^*T*^ are also symmetric matrices. According to the definition of symmetric matrices, it can be seen that

(16) $$\begin{array}{c} \text{tr}\left(ZBZ^{T}\right)=\text{tr}\left({\left(ZBZ^{T}\right)}^{T}\right), \end{array}$$

(17) $$\begin{array}{c} \text{tr}\left(ZAZ^{T}\right)=\text{tr}\left({\left(ZAZ^{\text{T}}\right)}^{T}\right), \end{array}$$

established.

The article "Classification of Artistic Styles of Chinese Art Paintings Based on the CNN Model" was published in 2022. Journal: Comput Intell Neurosci.

Substitute **Z** **=** **SP** and formulas (15) and (16) into formula (13); then

(18) $$\begin{array}{c} \underset{pp^{T}=1}{\text{min}}C_{\text{F}}=\underset{pp^{T}=1}{\text{min}}tr\left(ZBZ^{T}\right)\\ =\underset{pp^{T}=1}{\text{min}}tr\left(Z^{T}BZ\right)\\ =\underset{pp^{T}=1}{\text{min}}tr\left(P^{T}S^{T}BSP\right). \end{array}$$

Substitute *Z* = SP and formulas (16) and (17) into formula (14); then

(19) $$\begin{array}{c} \underset{pp^{T}=1}{\text{max}}D_{\text{E}}=\underset{\mathrm{pp}{=}^{T}1}{\text{max}}tr\left({\text{ZAZ}}^{T}\right)\\ =\underset{pp^{T}=1}{\text{max}}tr\left(Z^{T}AZ\right)\\ =\underset{pp^{T}=1}{\text{max}}tr\left(P^{T}S^{T}ASP\right). \end{array}$$

The optimal mapping matrix *P* is obtained by solving the formula (11) or (12). The experimental results show that although the mapping matrices obtained by solving formula (11) or (12) are different, the classification results of the datasets obtained after the mapping calculation are the same.

**Step 8 .**

Calculate the new training dataset **Z** and test dataset **Z**′ generated by the embedded mapping.

A new training dataset **Z** can be obtained by mapping the set **S** calculated in Step 6, and a new test dataset **Z**′ can be obtained by mapping the set **S**′, that is, **Z**=**SP**, **Z**′=**S**′**P**.

## 3. Experiments

The number of works created by Chinese painting writers in their lifetime is relatively small; therefore, compared with the classification of ordinary images, the amount of data on Chinese painting works is relatively small. At present, there is no standard dataset of Chinese paintings. Based on the above situation, the experimental dataset in this study contains 100 paintings of 10 Chinese painters from ancient times to the present, and 70% of the paintings are used as the training sample set. The remaining part is used as the test sample set, and the data in the training and test sample sets do not overlap. The ten painters are CDY, CSF, FZ, HYY, HZ, LDZ, LKL, TY, XBH, and BDSR. In this study, SVM [27–30] is used for classification experiments.

The article "Classification of Artistic Styles of Chinese Art Paintings Based on the CNN Model" was published in 2022. Journal: Comput Intell Neurosci.

To test the algorithm in this study, the experiments will be designed from the following four aspects: to verify the influence of the change in the number of painters on the classification accuracy, the classification experiment was conducted to compare the works of 5 painters and 10 painters, respectively; to verify the effectiveness of the algorithm, it is compared with the existing literature such as fusion, MHMM, and other algorithms; to verify the effectiveness of the feature extraction of the VGG-F model, the algorithm in this study is compared with the traditional feature extraction algorithms based on color (HSV), texture (Gabor), and shape (HOG); and to verify the impact of the embedded learning introducing mutual information on the classification, the algorithm in this study is compared with the DEFC algorithm and the pure SVM algorithm.

This study uses the precision rate P (precision) and the recall rate R (recall) to evaluate the execution results of the algorithm, which are defined as *P*=*a*/*a*+*b* and *R*=*a*/*N*, respectively. Among them, *a* is the number of samples that are correctly classified into this class, *b* is the number of samples that are wrongly classified into this class, and N is the number of samples of this class in the test dataset. Considering the first aspect, this study selects the works of 5 painters and 10 painters for experimental comparison, and the comparison results are shown in Tables 1 and 2. It can be seen that the increase in the number of painters has a certain impact on the classification results. The precision and recall rates of the MIDEC algorithm in this study are 94.88% and 87.49% in the classification of the two cases. Although the accuracy rate has decreased, the magnitude is not very large. The experimental results show that the algorithm in this study has certain robustness.

The algorithm in this study is compared with the fusion and MHMM algorithms experimentally. It can be seen from Tables 1 and 2 that the MIDEC algorithm in this study has the highest classification accuracy on the two sets of works; among them, the precision and recall rates of LKL and XBH's paintings are the highest because the two painters have unique painting styles. XBH's paintings are rough, vigorous, and majestic; they pay attention to the anatomical structure of the object, the accurate grasp of the bones, and pay great attention to the modeling. It has a swaying style that is unrestrained without being arrogant and subtle without being trivial; LKL perfectly reproduces the realistic spirit of Western painting with the tools and materials of Chinese painting. The works are slender and realistic, with a natural look. The art styles of the 2 painters differed the most from the other painters, resulting in the highest accuracy. It can be seen from Table 2 that the recall rate of HZ in this algorithm is 32.99%, which is the lowest recall rate among the 10 painters. This is because HZ copied paintings in the Forbidden City in Beijing for a long time, drawing on the strengths of many families, making his style unpredictable, resulting in a low recognition rate of paintings.

The article "Classification of Artistic Styles of Chinese Art Paintings Based on the CNN Model" was published in 2022. Journal: Comput Intell Neurosci.

As shown in Table 1, compared with the HSV + Gabor + HOG + MIDEC algorithm, the precision and recall of the algorithm in this study are increased by 17% and 18%, respectively. It is proved that the features extracted by the VGG-F model can more effectively reflect the different artistic styles of painters.

As shown in Table 1, the precision and recall of the algorithm in this study are higher than those of the pure SVM and DEFC algorithms, which prove that the introduction of mutual information and embedded can further improve the classification accuracy.

It is known from experiments that for Chinese paintings with different themes and styles that are similar in style and with the same theme and different styles, the algorithm in this study has good robustness in classification.

## 4. Conclusions

Most of the existing classifications of Chinese paintings only consider the correlation between paintings and class labels, ignoring the correlation between paintings and the influence of feature importance. In this study, the image features of Chinese painting are extracted by fine-tuning the pretrained VGG-F model. Based on the DEFC algorithm, the mutual information theory is introduced, and an embedded classification algorithm based on mutual information is proposed, which makes the embedded principle affected by feature selection and feature importance. Experiments show that this algorithm has strong robustness.

In addition to analyzing the style characteristics of the painting itself, the identification of Chinese painting painters should also include the analysis of paper color, ink color, color components, style identification, and seals Adding other factor analysis can help overcome the decline of recall and precision, which will be part of the future work. In addition, the existing image emotion research mainly focuses on natural images and face images, lacking the digital description system of Chinese painting emotion, so the next work will also be carried out on the emotional classification of Chinese painting.

The article "Classification of Artistic Styles of Chinese Art Paintings Based on the CNN Model" was published in 2022. Journal: Comput Intell Neurosci.

## Figures and Tables

**Table 1:** Comparison of the classification results of the works of five painters by different algorithms.

Painters	This paper algorithm		Fusion		MHMM		HSV + Gabor + HOG + MIDEC		DEFC		SVM	
	*P*	*R*	*P*	*R*	*P*	*R*	*P*	*R*	*P*	*R*	*P*	*R*
CDY	0.9023	0.9298	0.8323	0.7998	0.7923	0.7698	0.8223	0.8998	0.9023	0.8998	0.8923	0.8298
CSF	0.9296	0.9004	0.8096	0.8304	0.8296	0.8004	0.5996	0.7004	0.8196	0.9004	0.8496	0.9304
LKL	0.9423	0.9998	0.7923	0.7698	0.8423	0.8998	0.8423	0.8698	0.9023	0.8998	0.9623	0.7998
XBH	0.9696	1	0.8396	0.9004	0.8396	0.8704	0.7796	0.7004	0.9996	1	0.8796	0.9704
BDSR	1	0.8998	0.9023	0.8698	0.9023	0.8698	0.8823	0.6998	0.9623	0.8698	0.8723	0.8998
Mean	0.9488	0.9460	0.8352	0.8340	0.8412	0.8420	0.7852	0.7740	0.9172	0.9140	0.8912	0.8860

**Table 2:** Comparison of the classification results of 10 painters' works by different algorithms.

Painters	This study algorithm		Fusion		MHMM	
	*P*	*R*	*P*	*R*	*P*	*R*
CDY	0.8498	0.9302	0.7598	0.7302	0.7498	0.7002
CSF	0.8503	0.9299	0.7403	0.7699	0.7303	0.7299
FZ	0.7297	0.8997	0.7197	0.7697	0.7997	0.7997
HYY	0.6998	0.9302	0.7898	0.7702	0.7398	0.7702
HZ	0.9103	0.3299	0.5903	0.5299	0.6203	0.5999
LDZ	0.8697	0.8997	0.7197	0.6997	0.7397	0.7697
LKL	0.9698	0.9702	0.7298	0.7302	0.8098	0.8702
TY	0.9703	0.9699	0.7803	0.8299	0.8903	0.8299
XBH	0.9397	0.9997	0.8097	0.8697	0.8097	0.8297
BDSR	0.9598	0.7302	0.8598	0.8302	0.8298	0.8302
Mean	0.8749	0.8590	0.7499	0.7530	0.7719	0.7730

## Data Availability

The dataset used to support this study can be accessed upon request.
